# Adipose-Derived Mesenchymal Stem Cell-Derived Extracellular Vesicles Rescue Tendon Injury in Rat via the miR-19 a/IGFBP3 Axis

**DOI:** 10.1155/2022/4197473

**Published:** 2022-09-12

**Authors:** Haibo Zhao, Hongyuan Jiang, Haoyun Zhang, Zewen Sun, Qian Lin, Tianrui Wang, Tengbo Yu, Yingze Zhang

**Affiliations:** ^1^Department of Orthopedics, Qingdao University Hospital, Qingdao 266000, China; ^2^Trauma and Emergency Center, The Third Hospital of Hebei Medical University, Shijiazhuang 050051, China

## Abstract

**Purpose:**

Adipose-derived mesenchymal stem cells (ADSCs) are increasingly applied in tendon repair. However, the underlying mechanisms of ADSC-derived extracellular vesicles (EVs) in tendon healing are largely unknown. In this study, we investigated the effect of the EVs secreted by ADSCs on the recovery of tendon injuries and its potential mechanism.

**Materials and Methods:**

We injected ADSCs into the injured tendon, followed by the evaluation of the tissue morphology, tenocyte proliferation, and oxidative stress. Then, the injured tenocytes were treated with EVs secreted by ADSCs, and oxidative stress and proliferation of tenocytes *in vitro* were detected. After the overexpression and knockdown of miR-19a and its target protein IGFBP3, the oxidative stress and proliferation of tenocytes *in vitro* were assessed. Finally, the injured tendon was treated with EVs, and the tissue morphology and proliferation of the injured tendon *in vivo* were examined.

**Results:**

ADSC-derived EVs were found to inhibit oxidative stress and promote proliferation of tenocytes isolated from an injury model of rats. EVs were shown to carry miR-19a which regulated the expression of IGFBP3 through binding to 3′UTR of IGFBP3 mRNA. In addition, IGFBP3 promotes oxidative stress and inhibits proliferation of tenocytes. Finally, we found that ADSC-derived EVs promoted tendon wound healing *in vivo*.

**Conclusions:**

Our data suggest that treatment with ADSC-derived EVs ameliorates tendon injury by inhibiting oxidative stress and promoting proliferation in tenocytes. miR-19a carried by ADSC-derived EVs regulates IGFBP3 expression through binding to its 3′UTR.

## 1. Background

Tendons, a component of the musculoskeletal system, are the connective tissues that transmit force from muscles to bones [1]. Tendon injury, such as tendon rupture or tendinopathy, often occurs in sports or at workplaces [2]. Multiple strategies are available for the treatment of tendon injury, including conservative management (e.g., immobilization, physiotherapy programs, or nonsteroidal anti-inflammatory drugs) and surgical interventions, depending on the site and extent of the injury [3, 4]. These methods are sometimes accompanied by poor recovery or the potential harm of drugs to the patient's body (anti-inflammatory drugs, e.g., corticosteroid injections) [5, 6]. In recent years, mounting evidence has demonstrated that mesenchymal stem cells (MSCs) are involved in tissue repair. Further, MSCs derived from tendon or nontendon or adipose tissue have also received increasing attention in enhancing tendon healing. It has been suggested that MSCs can help accelerate and improve the quality of tendon healing *in vitro* and *in vivo* studies. However, the underlying mechanisms of MSCs in tendon repair are still largely unknown [7].

MSCs are adult stem cells derived from the mesoderm [8]. They have the potential for multidirectional differentiation, which forms the basis of potential treatment for numerous human diseases [9, 10]. MSCs secrete exosomes to repair the damaged tissues and restore tissues' function (e.g., tendon-bone healing, cutaneous wound healing) [11, 12]. It is implicated that MSCs improve tendon healing at least partly via a paracrine mechanism [13]. Extracellular vesicles (EVs) are nanometer-sized cell-secreted membrane vesicles. They contain biologically active substances and are secreted to the extracellular environment through the process of “endocytosis-fusion-efflux” from the intracellular multivesicles and cell membrane. EVs are formed and secreted by most cells, including MSCs, which can mediate information exchange among cells and regulate the functions of surrounding cells [14, 15]. EVs secreted by MSCs have the characteristics of low toxicity, easy extraction and preservation, and low possibility of immune rejection, which showed similar biological properties as MSCs [16]. EVs contain a large amount of noncoding RNAs, including miRNAs, which play an important role in MSC-mediated tissue recovery [17].

miRNA is a group of noncoding RNA with an average length of ~22 nucleotides that regulates biological functions through binding to mRNA 3′UTR. It is a key regulatory molecule in most physiological or pathological activities such as cell differentiation, cell proliferation, and cell apoptosis [18]. miR-19 is a member of the oncogenic miR-17-92 family and acts as a proliferation promoter in many cells. For example, it has been found to promote proliferation, invasion, and migration of osteosarcoma cells by inhibiting SPRED2-mediated autophagy [19]. In glioma cells, miR-19a has been reported to promote cell proliferation via the SEPT7-AKT-NF-*κ*B pathway. However, its role in tendon repair has not been reported to date [20].

In this study, we found that miR-19a was carried to tenocytes by MSC-EVs and promoted tendon repair by targeting 3′UTR of IGFBP3 in tenocytes.

## 2. Materials and Methods

### 2.1. Animal Experiments and Cell Culture

The healthy Sprague-Dawley (SD, Cyagen Biosciences, China) rats (12 weeks old, 300-330 g) were divided into three groups, and the rat tendons were cut off for one week. ADSCs (1 × 10^6^ cells per rat), and EVs secreted by ADSCs (50 *μ*g per rat) were injected into the injured tendons of rats in the injury+ADSC group and injury+EV group, respectively. After continuous injection once a day for 4 weeks, the rats were euthanized. The injured group was injected with the same volume of saline once a day for 4 weeks. Routine injection of penicillin was administered to prevent infection after operation. The tendons of the rats in the control group were not cut but injected with the same volume of saline same as the injury group.

The tenocytes, ADSCs (Percell, China), and 293T cells (Fenghbio, China) were cultured in Dulbecco's modified Eagle's medium (DMEM, Gibco BRL, USA) supplemented with 10% fetal bovine serum (FBS, Gibco, BRL, USA), 100 U/mL of penicillin, and 100 *μ*g/mL of streptomycin. Bone marrow-derived MSCs (BM-MSCs, Percell, China) were maintained in Ham's F12 medium (F12, Gibco, BRL, USA) supplemented with 10% FBS (Gibco, BRL, USA), 100 U/mL of penicillin, and 100 *μ*g/mL of streptomycin. ADSCs were selected for detection of the expression of stem cell surface markers ((cluster of differentiation (CD)45, CD34, CD29, and CD90 (all from Abcam, USA)) using flow cytometry (FCM). In addition, other ADSCs were induced to differentiate and stained with alizarin red (Cyagen Biosciences, USA), Oil Red O (Sigma-Aldrich, USA), and Alcian blue (Sigma-Aldrich, USA) to analyze the osteogenic, adipogenic, and chondrogenesis differentiation potential correspondingly. In cell experiments, ADSCs (1 × 10^4^ cells per plate) and tenocytes (1 × 10^5^ cells per plate) were cocultured as the injury+ADSC group (12-well plates, Corning, USA). Tenocytes (1 × 10^5^ cells per plate) were added with 10 *μ*g ADSCs-EVs (dissolved in 100 *μ*L PBS) as the injury+EV group. All cells were cultured in an atmosphere at 37°C with 5% CO_2_.

### 2.2. Flow Cytometry

The Annexin V-FITC/PI Apoptosis Detection Kit (BD Biosciences, USA) was used to analyze the apoptosis rate according to the instructions of the manufacturer. Briefly, the cells (4 × 10^5^ cells) were collected and resuspended. 5 *μ*L Annexin V-FITC and 5 *μ*L PI were added, and the cells were incubated for 25 min in the dark at room temperature. Cells were analyzed by FCM (BD FACSCanto, USA) within 1 h.

### 2.3. HE Staining

The paraffin sections were baked at 65°C for 30 min, dewaxed by xylene, dehydrated with gradient alcohol, washed with running water for 1 min, and then stained with HE. After washes under running water, sections were differentiated with 1% hydrochloric acid alcohol, followed by washes under running water. Then, the stained sections were dehydrated with alcohol, transparentized by xylene, and sealed with gum. Images were acquired on an Olympus BH2 microscope (Olympus Corporation, Japan).

### 2.4. Immunohistochemical Staining

Sections were deparaffinized and rehydrated, followed by antigen retrieval and incubation with 1% H_2_O_2_ in methanol for 15 min to block endogenous peroxidase. After being blocked with 5% bovine serum albumin, sections were incubated overnight with antibody (PCNA: Abcam, UK, 1 : 100; Caspase-3: Abcam, UK, 1 : 100) at 4°C. Then, they were incubated sequentially with a biotinylated secondary antibody and horseradish peroxidase-conjugated streptavidin (Abcam, USA, 1 : 800) for 30 min at 37°C. Immunoreactivity was visualized using diaminobenzidine (DAB). Then, a light hematoxylin counterstain was applied. Images were captured by an Olympus BX53 microscope (Olympus, Japan).

### 2.5. Enzyme-Linked Immunosorbent Assay (ELISA)

The levels of LDH (Yanjin, China), CK (Xitang, China), SOD (Chuangxiang, China), and MDA (Duma, China) in cell supernatant were measured using ELISA kits. The assay was conducted following the manufacturer's protocols. The OD value at 450 nm of each well was detected by Perlong a DNM-9602 Microplate Reader (China).

### 2.6. 3-[4,5-Dimethylthiazol-2-yl]-2,5 Diphenyl Tetrazolium Bromide (MTT) Assays

The cells were cultured in a 96-well plate at a concentration of 1 × 10^3^ cells/well. 20 *μ*L of 5 mg/mL MTT solution was added to each well and then cultured for 4 h. Afterwards, the culture medium was removed, and 150 *μ*L dimethyl sulphoxide was added to each well and incubated at 37°C with 5% CO_2_ for 10 min. The optical density (OD) value of each well at 490 nm was detected by a microplate reader. Three wells were used for each group.

### 2.7. Western Blot

Proteins were isolated in 200 *μ*L of RIPA buffer supplemented with protease and phosphatase inhibitors. The homogenates were cleared by centrifugation at 12,000 × g for 20 min at 4°C. Total protein concentration was evaluated using the BCA Protein Assay Reagent Kit (Beyotime, China). Protein samples were mixed with 6 × buffer. After boiling for 5 min, 30 *μ*g of proteins was loaded on a 10% or 12% sodium dodecyl sulphate polyacrylamide gel for protein separation and electrotransferred onto polyvinylidene fluoride membranes (Millipore, USA). Then, the membranes were blocked with 5% milk in TBST and incubated with the following diluted primary antibodies overnight at 4°C: the antibodies against PCNA (Abcam, UK, 1 : 1000), Caspase-3 (Abcam, UK, 1 : 1000) and the secondary antibodies (Abcam, UK, 1 : 8000). The gray value of each band was detected by chemiluminescence substrate, and the expression level of the target protein was expressed by the ratio of the gray value of the target band to the inner reference band (Boster, China).

### 2.8. Concentration and Identification of Exosomes

Based on the previous research [21, 22], when the cell density of the fourth-generation ADSCs and BM-MSCs reached 80%, the cells were observed under the microscope, and the EV-free medium (supplemented with EV-free FBS, System Biosciences, USA) was replaced for continuous culture for 48 h. The collected medium was centrifuged (at 300 × g for 10 min, 2,000 × g for 10 min, and 10,000 × g for 30 min) to remove dead cells and cell debris. Afterwards, the supernatant was filtered through a 0.22 *μ*m membrane (Merck Millipore Ltd., Germany), followed by the placing of the supernatant in an ultracentrifuge at 100,000 × g for 90 min. Finally, the EVs were resuspended in 100 *μ*L PBS. In addition, Exosome Purification Kit (Norgen Biotek, Canada) also was used to separate EVs. qRT-PCR was used to detect the expression level of miR-19a in EVs proposed by the two methods.

The morphology and ultrastructure of ADSCs-EVs were observed under the transmission electron microscope (TEM, HT-7700, Hitachi, Japan). Dynamic Light Scattering (DLS) was used to analyze the particle size of ADSCs-EVs (Instruments, Ltd., UK). According to a previous study, the expression of CD63 and TSG101 (Abcam, 1 : 1000, UK) was identified by Western blot.

### 2.9. Cell Coculture

Cell coculture was performed by the Transwell chamber (0.4 *μ*m, 12-well plates, Corning, USA). ADSCs were loaded in the upper chamber and cultured in serum-free medium. Tenocytes were loaded, seeded, and cultured in EV-free FBS medium (System Biosciences, USA) for 48 h.

### 2.10. Quantitative Real-Time Polymerase Chain Reaction (qRT-PCR)

Total RNA was isolated from tissues and cell lines using TRIzol reagent (TakaRa, Japan) and then reverse transcribed using the PrimeScript RT reagent Kit with gDNA Eraser (TakaRa, Japan). qRT-PCR was performed through the kit instructions of SYBR@ Premix Ex Taq™ II (TakaRa, Japan) on iQ5 Real-Time PCR System (Bio-Rad, USA). The results were normalized using GAPDH for mRNA or U6 for miRNA. Primers of the qRT-PCR were designed as shown in Table 1. Expression was calculated by the 2^-*ΔΔ*CT^ method. And all assays were performed in triplicate and independently repeated for three times.

### 2.11. Cell Transfection

The miR-19a mimics and ASO-miR-19a were synthesized by RiboBio (China). The overexpression plasmids of IGFBP3 (pcDNA3.1/IGFBP3) and si-IGFBP3 were synthesized by RiboBio (China). 20 nM of siRNA, mimics, and inhibitor of miR-19a or 4 *μ*g of plasmids was used to transfect tenocytes with Lipofectamine® 2000 (Thermo Fisher Scientific, Inc., USA) for 48 h in 6-well plates.

### 2.12. Luciferase Reporter Assays

The segments of wild-type IGFBP3 3′UTR containing the putative miR-19a binding sites (pmirGLO-IGFBP3 3′UTR wt) and mutant IGFBP3 3′UTR without the putative miR-19a binding sites (pmirGLO-IGFBP3 3′UTR mut) were synthesized and inserted into pmirGLO vectors. The pmirGLO-IGFBP3 3′UTR mut or pmirGLO-IGFBP3 3′UTR wt was cotransfected with miRNA mimic or NC into 293T cells. 48 h later, luciferase activity was detected using the Dual-Luciferase Reporter Assay System (Promega, USA).

### 2.13. Statistical Analysis

The GraphPad Prism 5 (GraphPad, USA) was used for data analysis. The data of experiments, which were performed at least three times and followed a normal distribution, are presented as mean ± standard deviation. The differences between groups were analyzed by Student's *t*-test for two groups and one-way analysis of variance (ANOVA) for three or more groups. *P* < 0.05 was considered statistically significant.

## 3. Results

### 3.1. Characterization of ADSCs

First, FCM was performed to measure the relevant biomarkers. As shown in Figure 1(a), CD29 and CD90 were highly expressed in ADSCs, while the expression level of CD34 and CD45 (hematopoietic cell markers) were not expressed in the ADSCs. Besides, the trilineage differentiation abilities of ADSCs was also tested. As shown in Figures 1(b)–1(d), ADSCs were differentiated to osteoblasts, adipocytes, and chondrocytes under induction medium.

### 3.2. ADSCs Rescued the Tendon Injury through Inhibiting Oxidative Stress and Promoting Proliferation in Tenocytes

In order to observe the effects of ADSCs on recovery of tendon injury, we established a tendon injury model and injected ADSCs into the injured site. HE staining showed that compared with the injury group, the collagen fibers of the tenocytes in the injured tendon treated with MSCs (injury+ADSC group) were arranged linearly in the same direction and more orderly (Figure 2(a)). Immunohistochemistry was used to detect the expression of PCNA and Caspase-3 in the control group, injury group, and injury+ADSC group. As shown in Figure 2(b), the expression of PCNA in the injury+ADSC group was higher than that in the injury group, but lower than that in the control group. By contrast, the expression of Caspase-3 in the injury+ADSC group was lower than that in the injury group, but higher than that in the control group. Then, we isolated three groups of tenocytes and performed ELISA to detect the expression of CK, LDH, MDA, and SOD in these cells. As shown in Figures 2(c)–2(f), the expression levels of CK, LDH, and MDA were lower in the injury+ADSC group than in the injury group. The expression level of SOD was higher in the injury+ADSC group than in the injury group. To further investigate the effect of bone marrow of ADSC on the recovery of tendon injury, MTT indicated that the activity of tenocytes in the injury+ADSC group cells was higher than that in the injury group cells, but lower than that in the control group cells (Figure 2(g)). FCM revealed that apoptosis of cells in the injury+ADSC group was reduced, as compared with that in the injury group (Figure 2(h)). PCNA is an essential factor in DNA replication and repair [23], and Caspase-3 is an apoptosis marker protein [24]. Then, we detected the relative expression levels of PCNA and Caspase-3 in those three groups by Western blot. The results showed an increase in the relative protein expression levels of PCNA and a decrease in the relative protein expression levels of Caspase-3 in the injury+ADSC group, as compared with the injury group. Conversely, compared with the control group, the relative protein expression level of PCNA in the injury+ADSC group reduced, while the relative protein expression level of Caspase-3 increased (Figure 2(i)). Collectively, these results suggested that ADSCs rescued the tendon injury through inhibiting oxidative stress and promoting proliferation in tenocytes.

### 3.3. ADSC-Derived EVs Inhibited Oxidative Stress and Promoted Proliferation of Tenocytes

To further detect the mechanism of phenotype changes in tendon injury treated with ADSCs, we purified exosomes secreted by ADSCs and detected their roles on the recovery of tendon injury. Firstly, we observed the structure and markers of exosomes using TEM, DLS, and Western blot, respectively. TEM results presented flat exosomes and a double-sided concave structure, with a diameter of 40-120 nm (Figure 3(a)). DLS results showed that the particle size of exosomes mainly concentrated between 100 and 200 nm. (Figure 3(b)). The marker proteins CD9 and TSG101 of exosomes were detected by Western blot (Figure 3(c)). Secondly, we incubated tenocytes isolated from injured tendon with EVs secreted by ADSCs (injury+EVs). As shown in Figures 2(d)–2(g), the expression levels of CK, LDH, and MDA were lower in the injury+EV group than in the injury group, while the SOD expression level was higher than that in the injury group, indicating that exosomes reduced the oxidative stress. MTT showed that the activity of tenocytes was higher in the injury+EV group than in the injury group (Figure 3(h)). We also found that the apoptosis of cells in the injury+EV group was reduced, as compared with that in the injury group (Figure 3(i)). Finally, we detected the relative expression levels of PCNA and Caspase-3 in those three groups by Western blot. The results displayed that compared with the injury group, the relative expression levels of PCNA in the injury+EV group increased, while the relative protein expression levels of Caspase-3 decreased (Figure 3(j)). These data indicated that ADSC-secreted EVs could resist oxidative stress and promote proliferation in tenocytes.

### 3.4. miR-19a Inhibited Oxidative Stress and Promoted Proliferation of Tenocytes

In order to explore the mechanism of the substance carried by exosomes in tendon injury recovery, literature review found that miR-19a could rescue cell injury [25, 26]. We used high-speed differential centrifugation and Exosome Purification Kit to compare the expression levels of miR-19a in EVs between different groups. As shown in Figures 4(a)–4(d), miR-19a expression was found in both ADSCs-EVS and BM-MSCs-EVs proposed by the two methods. And we found that the relative expression of miR-19a was higher in both the injury+ADSC and injury+EV groups than in the injury group (Figure 4(e)). We next analyzed the effects of miR-19a on tenocytes isolated from tendon repair. ELISA revealed that miR-19a could significantly reduce the expression levels of CK, LDH, and MDA in tenocytes and increase SOD level (Figures 4(f)–4(i)). MTT showed that overexpression of miR-19a promoted the activity of tenocytes (Figure 4(j)). FCM indicated that overexpression of miR-19a inhibited apoptosis of tenocytes isolated from injured tendon (Figure 4(k)). Subsequently, we detected the relative expression levels of PCNA and Caspase-3 by Western bolt. As shown in Figure 4(l), overexpression of miR-19a promoted the expression of PCNA and inhibited the expression of Caspase-3. Conversely, the expression levels of PCNA reduced after miR-19a was inhibited, while the expression levels of Caspase-3 increased. These results indicated that miR-19a carried by EVs inhibited oxidative stress and promoted proliferation in tenocytes.

### 3.5. EV-Derived miR-19a Inhibited IGFBP3 Expression through Targeting Its 3′UTR

We used DIANA-LncBase V2 and Targetscan to predict that IGFBP3 3′UTR had putative binding sites of miR-19a (Figure 5(a)). To verify this prediction, we cotransfected pmirGLO-IGFBP3-3′UTR wt with miR-19a mimics, ASO-miR-19a, or their corresponding control and found that overexpression of miR-19a decreased, whereas inhibition of miR-19a increased the relative luciferase activity significantly; these alterations were abolished when 293T cells were cotransfected with pmirGLO-IGFBP3 3′UTR mut with miR-19a mimics, ASO-miR-19a, or their corresponding control (Figure 5(b)). In addition, we used qRT-PCR to detect the relative expression of IGFBP3 after overexpressing or inhibiting miR-19a and found that overexpression of miR-19a could significantly decrease the relative expression of IGFBP3 in tenocytes. Conversely, inhibition of miR-19a significantly increased the relative expression of IGFBP3 in tenocytes (Figure 5(c)). Finally, qRT-PCR found that the relative expression of IGFBP3 mRNA level was lower in both the injury+ADSC and injury+EV groups than in the injury group (Figure 5(d)). These data indicated that miR-19a could negatively regulate IGFBP3 expression by targeting its 3′UTR.

### 3.6. IGFBP3 Promoted Oxidative Stress and Inhibited Proliferation of Tenocytes

Then, we analyzed the effects of IGFBP3 on oxidative stress and proliferation of tenocytes. As shown in Figures 6(a)–6(d), IGFBP3 decreased the SOD level and increased CK, LDH, and MDA levels in tenocytes. MTT showed that IGFBP3 inhibited the activity of tenocytes (Figure 6(e)). FCM suggested that inhibition of IGFBP3 reduced apoptosis of tenocytes (Figure 6(f)). Western blot displayed that IGFBP3 inhibited the relative protein expression of PCNA and promoted the expression level of Caspase-3 (Figure 6(g)). These results suggested that the miR-19a/IGFBP3 axis inhibited oxidative stress and promoted proliferation in tenocytes.

### 3.7. EVs Promoted Tendon Wound Healing In Vivo

Finally, we injected the EVs secreted by ADSCs into the injured tendon of rats. HE staining displayed the disordered structure of the tendon tissue, a large number of infiltrated inflammatory cells, and formation of vacuoles in the injury group, as compared with the control group. Compared with the injury group, the injury+EV group had fewer infiltrated inflammatory cells and improved tissue structure, significantly reduced tissue vacuole and structural disorder, and presence of vacuoles (Figure 7(a)). The results of immunohistochemistry and Western blot showed that compared with the injury group, the relative protein expression levels of PCNA in the injury+EV group increased, while the relative protein expression level of Caspase-3 decreased (Figures 7(b) and 7(c)). These data highlighted the role of MSC-derived EVs in promoting tendon wound healing *in vivo*.

## 4. Discussion

Tendon injury occurs frequently during sports and other rigorous activities [2]. The naturally healed tendon often has inferior mechanical properties and is susceptible to reinjury [3, 4]. To date, functional healing of tendon injury has been a great challenge. Studies have shown that MSCs have high differentiation potential and exert protective and repair effects on injured tissues [27, 28]. In particular, the frequency and yield of ADSCs were much higher than those of BM-MSCs [29]. In this study, ADSCs were injected into the injured tendon tissue in rats, and it was found that compared with the injury group, the collagen fibers of the tenocytes were arranged linearly in the same direction and orderly. Meanwhile, the level of oxidative stress was reduced, and tenocyte proliferation ability was increased. Accordingly, we hypothesize that ADSCs are effective in the repair of tendon injury by inhibiting oxidative stress and promoting proliferation of tenocytes.

MSCs displayed its repair capacity on multiple mechanisms, including releasing cytokines, expressing growth factors, and altering immune response [30]. In recent years, mounting evidences have revealed that MSCs perform their functions by paracrine mode. For example, MSCs release IL1RN to recover bleomycin- (BLM-) induced inflammation and fibrosis [31]. Li et al. reported that TGF-*β*1-containing exosomes derived from BM-MSCs could promote proliferation, migration, and fibrotic activity in rotator cuff tenocytes [32]. In this study, we confirmed that ADSCs secreted EVs using 3 methods. And we also found that EVs secreted by ADSCs could inhibit oxidative stress and promote proliferation of tenocytes, which displayed the same functions as ADSCs.

EVs carry various RNAs or proteins to the recipient cells to affect the functions of recipient cells. However, some studies suggest that high-speed separation methods lead to high contamination of EVs [33]. We used high-speed differential centrifugation and polymer precipitation to extract EVs from two types of MSCs, and the results confirmed that miR-19a expression was upregulated in EVs. And we found that both ADSCs and EVs could promote the expression of miR-19a in tenocytes. We also detected high expression of miR-19a in injured tenocytes (cocultured or with exosomes added.) miR-19a acts as a proliferation promotor in the process of proliferation in various types of cells [21, 22]. Zhu et al. reported that folic acid protected neural cells against aluminum-maltolate-induced apoptosis by preventing miR-19 downregulation [34]. miR-19 had a promotive effect in curcumin's regulation of the miR-19/PTEN/AKT/p53 axis to inhibit proliferation of bisphenol A-induced breast cancer cells [35]. Consistent with the above results, our research also showed that miR-19a can inhibit oxidative stress and promote proliferation of tenocytes. The selection of effective targeting RNA marked the beginning of the research on molecular mechanisms. In this study, we found that miR-19a target IGFBP3 promoted tenocyte proliferation. And the relative expression of IGFBP3 was lower in the injury+MSC group and the injury+EVs group than in the injury group. These results confirmed the role of the miR-19a/IGFBP3 axis in tendon repair.

IGFBP3 is a key member of the insulin-like growth factor family that plays a pivotal role in human growth and development. It is currently found that it is abnormally high in patients with colon cancer, prostate cancer, and oral squamous cell carcinoma [36, 37]. Silencing IGFBP3 can induce the migration and invasion of endometrial cancer cells [38]. However, in other studies, it is believed that high expression of IGFBP3 can inhibit tumor proliferation and migration. Transfection of IGFBP3 with an overexpression plasmid can suppress the angiogenesis of head and neck squamous cells by inhibiting the production of vascular endothelial growth factor (VEGF) [39]. In this study, IGFBP3 promoted oxidative stress and apoptosis of tenocytes and reduced the activity of tenocytes. This might be related to the dual role of IGFBP3 in tumor cells. On the one hand, IGFBP3 could form a ternary complex with IGF to inhibit the mitogenic effect of IGF by ALS. On the other hand, IGFBP3 could effectively prolong the half-life of IGF by binding to IGF and increase the bioavailability of IGF in tissues. These two effects of IGFBP3 were regulated by a number of factors, which might be responsible for the inconsistent role of IGFBP3 in cell proliferation [40, 41]. Finally, we conducted animal experiments, and the results showed that after treatment with EVs, the vacuoles of damaged tenocytes were reduced, the cells were arranged relatively neatly, and the expression of proproliferation proteins increased. It was verified that ADSC-derived EVs promoted tendon wound healing *in vivo*.

The role of MSCs in tendon healing has received more and more attention and has been widely reported to enhance tendon healing, but the mechanism is not clearly elucidated [42]. Our study demonstrates the role of EVs secreted by ADSCs in promoting tenocyte proliferation and inhibiting oxidative stress, is beneficial to tendon healing, and proposes an important role of the miR-19a/IGFBP3 axis in the process.

However, there are limitations in the study. This study simply tested the effects of ADSCs and EVs on oxidative stress and tenocyte proliferation *in vitro* but did not detect the biomechanical properties of ADSCs and EVs on tenocytes. Furthermore, the effects of EVs from other non-adipose tissue-derived MSCs on the miR-19a/IGFBP3 axis in tenocytes and tendon injury animal models were not observed.

## 5. Conclusion

In conclusion, our study confirmed that miR-19a in EVs secreted by ADSCs promoted the repair of tendon injury through the miR-19a/IGFBP3 axis.

## Figures and Tables

**Figure 1:** Characterization of ADSCs. (a) The expression of biomarkers (CD29, CD34, CD45, and CD90) was detected by FCM. (b–d) Trilineage differentiation of ADSCs. (b) Osteoblast, base magnification: ×200; (c) adipocytes, base magnification: ×400; (d) chondrocytes, base magnification: ×200.

**Figure 2:** ADSCs rescued the tendon repair through inhibiting oxidative stress and promoting proliferation of tendon cells. (a) HE staining was performed in the control group, injury group, and injury+ADSC group (base magnification: ×200). (b) Immunohistochemistry detected the expression of PCNA and Caspase-3 in tendon tissues (base magnification: ×400). (c–f) ELISA was used to detect the levels of CK, LDH, MDA, and SOD in the control group, injury group, and injury+ADSC group. (g) MTT assay was conducted to detect the activity of tendons cells in the control group, injury group, and injury+ADSC group. (h) FCM was used to detect the apoptosis of cells. (i) The expression of apoptosis-related proteins was detected by Western blot (^∗^*P* < 0.05, ^∗∗^*P* < 0.01).

**Figure 3:** ADSC-derived EVs inhibited oxidative stress and promoted proliferation of tendon cells. (a) TEM was used to observe the structure of EVs (scale: 100 nm). (b) DLS was used to observe the particle size of EVs. (c) Western blot was used to detect the markers of EVs. (d–g) ELISA was used to detect the levels of CK, LDH, MDA, and SOD in the control group, injury group, and injury+EVs group. (h) MTT was used to detect the activity of tendon cells. (i) FCM for the detection of the apoptosis of tendon cells. (j) The expression of apoptosis-related proteins was detected by Western blot (^∗^*P* < 0.05, ^∗∗^*P* < 0.01, and ^∗∗∗^*P* < 0.001).

**Figure 4:** Effects of miR-19a on oxidative stress and proliferation of tenocytes. (a–d) qRT-PCR was used to detect the expression of miR-19a in EVs. (a, b) Detect EVs obtained by high-speed differential centrifugation. (c, d) Detect EVs obtained by Exosome Purification Kit. (e) qRT-PCR was used to detect the expression of miR-19a in exosomes secreted from tendon tissues. (f–i) ELISA was used to detect the levels of CK, LDH, MDA, and SOD both in the NC mimic group, miR-19a mimic group, ASO-NC group, and ASO-miR-19a group. (j) MTT was used to detect the activity of tenocytes. (k) FCM was performed to detect the apoptosis of tenocytes. (l) The expression of apoptosis-related proteins was detected by Western blot in the NC mimic group, miR-19a mimic group, ASO-NC group, and ASO-miR-19a group (^∗^*P* < 0.05, ^∗∗^*P* < 0.01, and ^∗∗∗^*P* < 0.001).

**Figure 5:** EV-derived miR-19a inhibited IGFBP3 expression through targeting its 3′UTR. (a) Putative binding sites of miR-19a and IGFBP3 mRNA 3′UTR were predicted by DIANA-LncBase V2 and Targetscan. (b) Luciferase reporter analysis was performed to detect the bindings between miR-19a and IGFBP3 in tendon cells. (c) The effect of miR-19a intervention on the expression of IGFBP3 in tendon cells was evaluated using qRT-PCR. (d) The expression of IGFBP3 was evaluated using qRT-PCR in the injury group, injury+ADSCs, and injury+EV groups (^∗^*P* < 0.05, ^∗∗^*P* < 0.01, and ^∗∗∗^*P* < 0.001).

**Figure 6:** IGFBP3 promoted oxidative stress and inhibited proliferation of tenocytes. (a–d) ELISA was used to detect the levels of CK, LDH, MDA, and SOD in the pcDNA3.1 group, pcDNA3.1/IGFBP3 group, si-NC group, and si-IGFBP3 group. (e) MTT was used to detect the activity of tendon cells in the pcDNA3.1 group, pcDNA3.1/IGFBP3 group, si-NC group, and si-IGFBP3 group. (f) FCM was performed to detect the apoptosis of tenocytes. (g) The expression of apoptosis-related proteins was detected by Western blot in the pcDNA3.1 group, pcDNA3.1/IGFBP3 group, si-NC group, and si-IGFBP3 group (^∗^*P* < 0.05, ^∗∗^*P* < 0.01, and ^∗∗∗^*P* < 0.001).

**Figure 7:** EVs rescued the tendon repair through promoting proliferation of tendon cells. (a) HE staining was used to detect tendon tissue. Base magnification: ×200. (b) Immunohistochemistry was performed to detect the expression of both PCNA and Caspase-3 in the tendon tissue. Base magnification: ×400. (c) The expression of apoptosis-related proteins was detected by Western blot in the control group, injury group, and injury+EV group (^∗^*P* < 0.05, ^∗∗^*P* < 0.01).

**Table 1:** Primer sequence.

Gene	Forward (5′-3′)	Reverse (5′-3′)
GADPH	CGCCAAATTTCTCCCCTGAA	CCGTAGTGCTGGGCAATGTTC
U6	GTGCAGGGTCCGAGGT	CTCGCTTCGGCAGCACA
miR-19a	GGGTGTGCAAATCCATGC	AACTGGTGTCGTGGAGTCGGC
IGFBP3	GTGCTCCACTTCGCTCCATC	CCACAGCGCTCCGTGTAG

## Data Availability

All data generated or analyzed during this study are included in this published article.
